# Impact of four different recumbencies on the distribution of ventilation in conscious or anaesthetized spontaneously breathing beagle dogs: An electrical impedance tomography study

**DOI:** 10.1371/journal.pone.0183340

**Published:** 2017-09-18

**Authors:** Tamas D. Ambrisko, Johannes P. Schramel, Ulrike Auer, Yves P. S. Moens

**Affiliations:** Anaesthesiology and Perioperative Intensive-Care Medicine, Department for Companion Animals and Horses, University of Veterinary Medicine, Vienna, Austria; University of Bari, ITALY

## Abstract

The aim was to examine the effects of recumbency and anaesthesia on distribution of ventilation in beagle dogs using Electrical Impedance Tomography (EIT). Nine healthy beagle dogs, aging 3.7±1.7 (mean±SD) years and weighing 16.3±1.6 kg, received a series of treatments in a fixed order on a single occasion. Conscious dogs were positioned in right lateral recumbency (RLR) and equipped with 32 EIT electrodes around the thorax. Following five minutes of equilibration, two minutes of EIT recordings were made in each recumbency in the following order: RLR, dorsal (DR), left (LLR) and sternal (SR). The dogs were then positioned in RLR, premedicated (medetomidine 0.01, midazolam 0.1, butorphanol 0.1 mg kg^-1^ iv) and pre-oxygenated. Fifteen minutes later anaesthesia was induced with 1 mg kg^-1^ propofol iv and maintained with propofol infusion (0.1–0.2 mg kg^-1^ minute^-1^ iv). After induction, the animals were intubated and allowed to breathe spontaneously (FIO_2_ = 1). Recordings of EIT were performed again in four recumbencies similarly to conscious state. Centre of ventilation (COV) and global inhomogeneity (GI) index were calculated from the functional EIT images. Repeated-measures ANOVA and Bonferroni tests were used for statistical analysis (*p* < 0.05). None of the variables changed in the conscious state. During anaesthesia left-to-right COV increased from 46.8±2.8% in DR to 49.8±2.9% in SR indicating a right shift, and ventral-to-dorsal COV increased from 49.8±1.7% in DR to 51.8±1.1% in LLR indicating a dorsal shift in distribution of ventilation. Recumbency affected distribution of ventilation in anaesthetized but not in conscious dogs. This can be related to loss of respiratory muscle tone (e.g. diaphragm) and changes in thoracic shape. Changing position of thoraco-abdominal organs under the EIT belt should be considered as alternative explanation of these findings.

## Introduction

The distribution of ventilation is a main determinant of ventilation and perfusion matching and the oxygenation of arterial blood [1]. However, information about the regional distribution of ventilation is difficult to obtain and most of these techniques (e.g. using fluorescent microspheres, scintigraphy and computed tomography (CT)) are invasive and/or result in radiation exposure. Electrical impedance tomography (EIT) may offer advantages because it is a non-invasive, radiation-free, easily applicable and repeatable method for examining the distribution of ventilation [2–4]. A disadvantage of EIT over the other methods is that it cannot measure total lung volume, therefore ventilation per unit of lung volume cannot be obtained by EIT alone. This method measures total changes in regional air content that is consistent with regional distribution of tidal volume (hereinafter “distribution of ventilation”). The fact that this information is obtained non-invasively and continuously suggests that EIT may have a huge potential as a monitoring tool for ventilated patients in the ICU [5] or during operations. In spite of the fact, that canine patients are also being ventilated in ICU [6] with a variety of lung conditions and they would potentially benefit from lung monitoring with EIT, it is not yet a common technique in veterinary medicine.

Clinically meaningful publications about the use of EIT in dogs are scarce. A 32 electrode EIT system has been used for detection of experimentally induced lung oedema [7], and a custom-made EIT device using 16 electrodes was favourably evaluated for measuring changes in lung air and liquid volumes [8] and lung hyperinflation [9] in anaesthetized dogs. A recent study showed good correlation of EIT and CT images in anaesthetized dogs which were ventilated at different PEEP levels [10]. These studies suggest that EIT may be useful in this species in an ICU setting. Nevertheless, the effects of anaesthesia and body positioning on EIT assessed distribution of ventilation would be important to document in dogs too because these factors commonly affect ventilated ICU patients. Therefore, the aim of this study was to examine these effects in beagle dogs.

## Materials and methods

### Animals

The experimental protocol was approved by the institutional ethics committee of the University of Veterinary Medicine Vienna and the national authority according to § 8ff of Law for Animal Experiments, Tierversuchsgesetz–TVG 2012 (GZ 68205/0079-II/3b/2013). Nine healthy castrated male university owned beagle dogs were used. The dogs were housed on campus, fed dry commercial dog food ad libitum and had continuous access to both in-door and out-door facilities, the latter was enriched with different cage types and levels and different items. The dogs were living in little groups and walked by students daily on campus premises. The dogs were aging 3.7 ± 1.7 (mean ± SD) years and weighing 16.3 ± 1.6 kg were used. Routine haematological and biochemical blood examinations were performed before the study and were within normal limits. The dogs were fasted for 12 hours and water was withdrawn for 2 hours before the experiments. After the study the animals were placed back to the colony for use in subsequent non-invasive studies.

#### Study design

Nine beagle dogs were assigned to a single experimental group and each animal was used as its own control (within-subject experiment).

Sample size calculations (SigmaPlot for Windows Version 11.0, Systat Software, San Jose, California, USA) indicated that 2 subjects would be sufficient to demonstrate expected changes (1.8 ± 0.4) in left-to-right Centre of Ventilation (COV) assuming α = 0.05 and β = 0.2. Data used for this calculation were extracted from a rat study [11].

### Experimental setup

The experiment started at the radiology building. A 20 g catheter was placed in the cephalic vein. A sham EIT electrode belt (containing 32 electrodes) was placed around the thorax of conscious dogs at the level of the apex beat of the heart. This position was also used for the real EIT belt and it was chosen because reviewing anatomical drawings and CT images of dogs revealed that thoracic cross sections at the level of cardiac apex contained the most lung tissue. This corresponds to the ideal EIT belt placement in dogs according to another study [12]. The sham EIT electrodes were not connected to an EIT device because the connecting wires would have adversely affected the radiographic images. The dogs were positioned in right lateral recumbency (RLR) and rested for 10 minutes. Thoracic radiographs were taken in RLR and dorsal recumbency (DR) then the dogs were turned back to RLR and the sham belts were removed. The animals then were transported to another building where the rest of the experiment was undertaken. The transportation took about 10 minutes.

A custom made EIT electrode belt (containing 32 electrodes) was placed around the thorax of conscious dogs in a similar position where the sham belt was applied before. The electrodes were mounted equidistantly on a rubber belt. A single electrode consisted of 4 x 4 gold plated blunt pins (each pin was 0.5 x 0.5 mm wide) arranged in 2 mm distances forming a square of 6 x 6 mm (Fig 1A). The pins had sufficient length (3.7 mm) to reach through the hair coat to the skin to safeguard a low impedance electrode-skin contact. The electrodes did not cause discomfort to conscious dogs because the animals did not oppose being positioned into different recumbencies and sometimes even fell asleep without any medication during the measurements (Fig 1B). The electrodes did not leave behind any mark on the skin. Contact resistance was minimized by using electrode gel (Henry Schein, Melville, NY, USA). Each of these electrodes was connected with cables to an EIT device (model DX 1800, Timpel [former Dixtal], Sao Paulo, Brazil). Detailed description of this system is available elsewhere [13]. Electrocardiographic electrodes were also attached to the dogs (Einthoven II.). The EIT data was downloaded and saved on a dedicated computer at 50 Hz sampling frequency.

**Fig 1:** Custom made EIT electrode belt with 32 electrodes. (A) Each electrode comprised of 4 x 4 gold plated blunt pins with sufficient length to reach through the hair coat. (B) The electrodes did not cause any discomfort to conscious dogs.

### Measurements in conscious dogs

Since the start of the experiment until this point the dogs were mostly lying in RLR position. After the setup was complete, the animals were allowed to rest for five minutes. This was followed by two minutes of EIT recording while still in RLR. Then the dogs were gently turned into DR, followed by left lateral (LLR) and sternal recumbencies (SR). The rest-measurement cycle was repeated in each recumbency; then the animals were turned back to RLR again.

### Anaesthesia

In order to establish a baseline before anaesthesia, another rest-measurement cycle was performed in RLR. This was followed by a slow (over 30 seconds) iv injection of a mixture of medetomidine (Domitor, Pfizer Animal Health BV, Capell a/d Ijssel, The Netherlands) 0.01, midazolam (Mayrhofer Pharmazeutika, Linz, Austria) 0.1 and butorphanol (Alvegesic, Alvetra u. Werfft, Wien, Austria) 0.1 mg kg^-1^. After the dogs became sedate 100% O_2_ was applied via a tight fitting face mask using a Bain breathing system and high (5–6 L minute^-1^) O_2_ flow. Fifteen minutes later 1 mg kg^-1^ propofol (Fresenius Kabi Austria GmbH, Graz, Austria) was injected slowly (over 60 seconds) iv. The tracheas of the dogs were intubated and the cuffs of the endotracheal tubes were inflated. During this process the lungs were not inflated manually to avoid an incidental alveolar recruitment. Propofol (0.1–0.2 mg kg^-1^ minute^-1^ iv) was infused for maintenance. Arterial blood pressure (via oscillometric method), arterial haemoglobin saturation of oxygen, end-tidal CO_2_, respiratory rate, heart rate and rhythm were monitored during anaesthesia (iPM-9800 patient monitor, Mindray, Shenzen, China) and the data were manually recorded in every five minutes. The plan was to abort procedure and provide supportive treatment to the animals if the mean arterial pressure or the arterial O_2_ saturation fell below 60 mmHg or 90%, respectively or any other condition developed that would be judged unsafe during clinical anaesthesia.

### Measurements in anaesthetized dogs

Another rest-measurement cycle was performed after induction of anaesthesia while the dogs were still lying in RLR. This was followed by turning the dogs to DR, LLR and SR and performing a rest-measurement cycle in each body position, similarly to conscious state. The dogs were turned back to RLR, the EIT belt was removed. The animals were transported back to the radiology building while still anaesthetized and the thoracic radiographs were repeated in RLR and DR. The experiment was terminated at this point and the animals were recovered in a routine manner.

### Post-hoc analysis of EIT data

A thoracic CT image of a beagle dog was used to create an EIT mesh for dogs. This mesh was used to create EIT video images while applying an intermediate Gaussian spatial filter and a low-pass temporal filter at 1 Hz (EIT Analysis Tools Beta 7.4.57, Timpel [former Dixtal], Sao Paulo, Brazil). Three similar breaths were selected from these video images near the end of each recording.

Two kinds of functional EIT images were created from each selection: SD images containing the pixel-wise standard deviations of the impedance signals and R images containing Pearson correlation coefficients (linear regression analysis of each pixel and a reference respiratory signal located in the middle of a lung).

During the analysis of SD images, only those pixel SD values were used where the R values were positive (respiratory signals). The following variables were calculated from each SD image: left-to-right and sternal-to-dorsal Centre of Ventilation (COV) [14], global inhomogeneity (GI) index [15]. Left-to-right COV expressed the distance from the left side of the thorax as % of the thoracic width and sternal-to-dorsal COV was the distance from the sternum as % of the thoracic height.

The GI indices were also calculated for the R images for the positive and the negative pixel R values separately. In case of negative R values, the GI indices were multiplied by -1. After the calculations were complete, the SD and R images were normalized and averaged across dogs. The Matlab software (version 7.7.0.471 (R2008b), MathWorks, Natick, MA, USA) was used for calculations.

### Statistical analysis

The following data were included in statistical analysis: left-to-right and sternal-to-dorsal COV and GI index. Normality of the data was examined with the Shapiro-Wilk test. The data were compared across recumbencies, for conscious and anaesthetized states separately, using RM-ANOVA with Greenhouse-Geisser corrections. If significance was found, Bonferroni test was used for multiple comparisons. These variables were also compared right before premedication (while in RLR) and after induction of anaesthesia (in RLR) using paired t-test. The test wise *p* value was less than 0.05 (SPSS, version 20, IBM, Armonk, NY, USA). Data is presented as mean ± SD.

## Results

Each of the nine dogs completed the study and maintained spontaneous ventilation without periods of apnoea. The averaged SD images show the distribution of ventilation in 4 recumbencies for both conscious and anaesthetized states (Fig 2). The averaged R images (Fig 3) contained only a few pixels that negatively correlated with ventilation (inverse respiratory signals). These signals were located at the sides of the images (blue colour) and did not seem to correspond to any particular anatomical structure (e.g. gas filled intestines).

**Fig 2:** Averaged functional EIT images showing the distribution of ventilation in nine beagle dogs in conscious and anaesthetized states in four recumbencies. The sequence of A to H represent the time course of the events. The arrows in the right lower corner indicate right and dorsal orientation of each EIT image. Pixel colour indicates intensity of ventilation (scale shows arbitrary units derived from SDs of ventilation signals). When animals were turned to LLR under anaesthesia the distribution of ventilation in the left lung shifted dorsally (compare image G to F) possibly because abdominal content protruded towards the left-sternal side of the thorax. In SR (under anaesthesia) the distribution of ventilation shifted right (compare image H to F) possibly because the pressure on the right lung (imposed by the abdominal content) decreased. Both changes were statistically significant (see Fig 4). RLR: right lateral recumbency, DR: dorsal recumbency, LLR: left lateral recumbency, SR: sternal recumbency.

**Fig 3:** Averaged functional EIT images showing the regression coefficient (Pearson R) for each pixel that significantly correlated with the reference respiratory signal. Pixels with red colour positively correlate with respiration (respiratory signals) but those with blue colour inversely correlate. Inverse respiratory signals occupy only a few pixels on the sides of the images and these are most likely artefacts. Unlike in horses, there is no indication that abdominal gas pockets would affect thoracic EIT images in dogs. See Fig 1 for more explanation.

The data were normally distributed. GI values did not change in this experiment (overall GI values were 0.35 ± 0.01). During conscious state there was no change in left-to-right (p = 0.074) and sternal-to-dorsal (p = 0.419) COV (Fig 4). Premedication, pre-oxygenation and induction of anaesthesia in RLR resulted in left and dorsal shifts in distribution of ventilation (Fig 5). Namely, left-to-right COV decreased (from 48.9 ± 2.6% to 47.2 ± 2.5%; *p* = 0.01) and sternal-to-dorsal COV increased (from 50.5 ± 1.1% to 52 ± 0.9%; *p* = 0.007). During anaesthesia both left-to-right (p = 0.008) and sternal-to-dorsal (p = 0.002) COV changed. Specifically, left-to-right COV increased (*p* = 0.03) from DR to SR (46.8 ± 2.8% and 49.8 ± 2.9%, respectively) indicating a right shift. Ventral-to-dorsal COV increased (*p* = 0.014) from DR to LLR (49.8 ± 1.7% and 51.8 ± 1.1%, respectively) indicating a dorsal shift in ventilation distribution. The changes in COV can be followed on the SD images (Fig 2).

**Fig 4:** **Mean (SD) of the left-to-right (A) and sternal-to-dorsal (B) centre of ventilation (COV) in conscious (open circles) and anaesthetized (closed circles) beagle dogs.** Abscissa indicates the recumbencies (see Fig 1). * indicate significant difference between values during anaesthesia.

**Fig 5:** **Averaged functional EIT images showing the distribution of ventilation right before premedication (A) and after induction of anaesthesia (B) in nine beagle dogs.** See Fig 2 for colour scale and image orientation. Note that Fig 5B image is identical to Fig 2E but Fig 5A was recorded after Fig 2D. Red arrows show the direction of change (left and dorsal) in distribution of ventilation after induction of anaesthesia. Thoracic Computed Tomography (CT) images (C and D) serve as anatomical reference. The CT images were recorded in a healthy beagle dog that was a clinical patient. The dog was anaesthetized and lying in sternal recumbency during CT examination. Image (C), containing the shadow of the heart, was taken 10 mm cranially from image (D), containing the shadow of the abdominal content. The distribution of lung fields on the CT images are similar to those of the EIT images above them. This observation suggests an alternative explanation for the EIT findings since induction of anaesthesia is likely to cause reduction of lung volume and cephalad displacement of the diaphragm. H: shadow of the heart, Abd: shadow of abdominal content, R: right.

Thoracic radiographs did not reveal signs of atelectasis development. The position of the sham EIT belt was ranging from the cardiac apex to mid cardiac area among the dogs and there were also differences within the same animal between recumbencies (Fig 6).

**Fig 6:** **Thoracic radiographs of a conscious beagle dog in right lateral (A) and dorsal (B) recumbencies before the experiment.** A sham EIT belt, containing metal electrodes, was placed around the thorax at the level of the punctum maximum of the cardiac apex beat. Note that placing the dog in dorsal recumbency and pulling the front legs forward resulted in a cranial shift in the position of the EIT belt in this case. Reviewing similar x-ray images of all the 9 dogs in this study revealed that the position of the sham EIT belt ranged from the level of the cardiac apex to mid cardiac area in lateral recumbency. R: right side.

## Discussion

Body position did not affect distribution of ventilation in conscious beagles. Sedation, pre-oxygenation and induction of anaesthesia in RLR caused left and dorsal shifts in distribution of ventilation. This may be explained by developing atelectasis in the right (dependent) lung areas and also by cephalad movement of the diaphragm. As the respiratory muscles relax during anaesthesia, the diaphragm may be bulging more into the sternal and dependent (right) areas of the thorax, possibly causing shifts in lung tissue in the opposite directions. When animals were turned to LLR under anaesthesia the distribution of ventilation on the left side of the thorax shifted dorsally (Fig 2G) possibly because of developing atelectasis on the left side and also abdominal content may have protruded cranially towards the left-sternal side of the thorax. Subsequently, in SR (under anaesthesia) the distribution of ventilation shifted right (Fig 2H) possibly because the pressure on the right lung (imposed by the abdominal content) decreased and therefore, the right lung was able to inflate more.

Changes in distribution of ventilation detected in this study can be explained by two mechanisms. One of them being atelectasis development and consequential changes in distribution of ventilation per unit of lung volume. And the other is the displacement of lung tissue under the EIT electrode belt because of possible cephalad movement of the diaphragm. This suspicion is supported by the fact that adjacent CT images (Fig 5C and 5D) showed substantial differences in distribution of aerated lung fields. These two mechanism are indistinguishable in this study but they are not mutually exclusive because compression by the protruding abdominal content may cause atelectasis. The fact that possible development of pulmonary atelectasis in this study could not be confirmed by radiographic images does not preclude atelectasis as possible explanation of the findings because thoracic radiography has poor sensitivity in detecting this condition [16,17].

The results of studies that report distribution of ventilation per unit of lung volume [18,19] are not directly comparable to those presented here. Similarly to the present findings, a study on spontaneously breathing non-anaesthetized human infants and adults found centrally positioned COV values that were unaffected by dorsal and sternal recumbencies [20]. However, the subtle changes in COV detected here are very different from those reported in anaesthetized rats [11] where large shifts were shown towards the non-dependent lung areas in each body position. A possible explanation for these differences may be that the rats were ventilated but the beagles were spontaneously breathing. Similar effect of mechanical ventilation was shown in dorsally recumbent horses, where COV moved towards the non-dependent area after initiating ventilation [21]. If mechanical ventilation had such an influence on distribution of ventilation it may enhance recumbency related differences in COV. However, this hypothesis need to be tested in dogs.

The existence of inverse respiratory signals is known [22] and a previous horse study from our institution demonstrated that the location of such signals was predictable and corresponded to the location of abdominal gas pockets [23]. Nevertheless, in the current study, the inverse signals were unremarkable and did not seem to correspond to any particular anatomical structure. Therefore, these are most likely artefacts caused by movement of the EIT electrodes during breathing [22,24] or by the reconstruction algorithm [25].

The pin equipped EIT electrode belt was well tolerated by the dogs and high quality EIT signals could be obtained. The fact that shaving the dogs may not be necessary when using such a belt may make it easier to recruit clinical patients for EIT monitoring projects.

A limitation of the study is that the variability of EIT electrode belt location and possible belt movement during rotation of animals may result in imaging slightly different thoracic segments among animals and treatments. This effect may contribute to the uncertainty of the measurements.

Another limitation is that the order of body positions were not randomised, therefore, position and the order of positions (e.g. lung volume history) may both affect the results. Randomization could be used to cancel out the effects of treatment order on the results at the expense of increasing random background noise. This technique only makes sense if the treatment effect is much larger than the treatment order effect so that the signal-to-noise ratio can be maintained. In this study it was decided not to randomize because the results of a pilot study indicated that recumbency during induction of anaesthesia may have large carry-over effect on subsequent EIT images possibly as a result of persistent atelectasis. Whether atelectasis would change after repositioning anaesthetized dogs was unknown for the authors but it was suspected that without an alveolar recruitment manoeuvre [26,27] atelectasis may not resolve quickly by changing body position.

## Conclusions

The combined effect of sedation, pre-oxygenation and induction of anaesthesia changed distribution of ventilation in a way that is consistent with development of pulmonary atelectasis. Further changes in distribution of ventilation were detected while changing recumbency during anaesthesia but not in conscious dogs, suggesting, that anaesthesia opposed the maintenance of distribution of ventilation. These changes may also be related to loss of respiratory muscle tone and subsequent displacement of lung tissue and abdominal content.

## Supporting information

S1 Table Experimental data. These are the COV and GI data collected during the study.
(XLSX)

S2 Table Statistical results. This is a summary of the statistical results.
(XLSX)

S1 Text ARRIVE checklist. This is the completed ARRIVE Checklist.
(PDF)
